# Presence of Contagious Bacterial Flora in Formalin-Fixed Cadavers: A Potential Health Hazard to Medical Professionals

This article has been retracted.

**DOI:** 10.7759/cureus.30684

**Published:** 2022-10-25

**Authors:** Ppavani Gundreddy, Sagar S Gaurkar

**Affiliations:** 1 Anatomy, Jawaharlal Nehru Medical College, Datta Meghe Institute of Medical Sciences, Wardha, IND; 2 Otolaryngology - Head and Neck Surgery and Surgical Oncology, Jawaharlal Nehru Medical College, Datta Meghe Institue of Medical Sciences, Wardha, IND

**Keywords:** formalin, disinfection, bacteria, dissection halls, cadavers

## Abstract

Cadaveric dissection is the most important learning tool in anatomy. Although many new modalities are coming up for learning anatomy, cadaveric dissection outstands all of these as it helps students to visualize the human body and remains the most realistic way of learning anatomy. The cadavers are preserved using formalin, a potent disinfectant. Even after embalming in 5-10% formalin, the cadaver might still be infectious while using it in the dissection hall (anatomy department). Numerous bacterial species and infectious pathogens might still be seen despite using fixative agents. Several disease-causing agents may remain viable. Earlier reports suggest that there are cases where students and the working staff got infected by HIV, viral hepatitis, tuberculosis, and prion diseases.

The main objective of this study is to determine if bacterial species could be recovered from cadavers that are formalin-fixed. Specific regions in the body such as the axilla, perineum, finger clefts, and oral and nasal cavities were chosen for microbiological examination to detect bacterial species. The presence of skin folds in these regions makes them potential sites for the growth of bacteria.

Formalin-fixed cadavers can still act as regions for the growth of viable bacteria that can be pathogenic and affect the health of students and anatomists handling them. Proper care should be taken regarding this because students and anatomists working with these cadavers may get exposed to pathogenic organisms which may become harmful or sometimes life-threatening. Some precautions for proper dissemination of cadavers should be taken to provide a complete, safe, and healthy ambiance in the dissection hall.

## Introduction and background

Cadavers have been one of the best tools to learn human anatomy for centuries. They help students learn about muscles, bones, vessels, and every minute structure of the human body in a very detailed manner [1]. This gives them more accurate knowledge about the size and location of every organ inside the body. Learning with the help of a cadaver teaches teamwork as a group of students works together at dissection hall tables helping out each other [2]. Cadaveric dissection makes anatomy more interesting and creates enthusiasm among students. The most common source of cadavers in dissection halls are unclaimed bodies or donated bodies of individuals. A few anatomists also import cadavers from other countries to conduct a variety of studies [3,4]. The cadavers have to be checked for the presence of microorganisms before handling them to students in the dissection hall. The main reason for embalming is to inhibit the growth of microorganisms and preserve the tissue for longer studies [5,6]. The commonly used embalming fluids include formalin, ethanol, and phenol, which are effective against infective agents such as bacteria, fungi, and spores. Formalin is an aqueous solution of formaldehyde that acts by the formation of covalent bonds, thus inhibiting the growth of various bacteria and fungi. Few studies indicate formalin being ineffective in removing all microorganisms from the surface of cadavers, while few show differences in the usage of formalin percentage that would affect the growth of microorganisms completely [7-9]. There are numerous viable organisms which include bacteria (*Staphylococci*, *Streptococci*, etc.) fungi (*Penicillium*, *Aspergillus*, etc.), and viruses present on formalin-fixed cadavers that can contaminate the dissection halls and transmit various diseases to students if proper care is not taken. They may transmit diseases such as HIV, hepatitis B and C, and tuberculosis to people handling cadavers in the dissection hall [10,11]. Proper protective clothing, maintenance of hygiene, vaccination against diseases such as hepatitis and tuberculosis to all those who handle cadavers, and staying up to date on the most recent literature in the field would be of great help to ensure safety [12,13]. This study would give us adequate knowledge: (1) to check for the presence of bacteria on formalin-fixed cadavers and determine whether they are commensal or pathogenic; and (2) to prevent anatomists and students from getting exposed to pathogenic organisms while handling the cadavers.

## Review

Common risk factors and their adverse effects

Chemicals

Formalin is the most commonly used chemical substance to preserve cadavers according to our regular practices. This is found to show various adverse effects on the students and dissectors which include headache, nausea, dizziness, dryness of eyes and mucous membranes, overflow of tears, and a burning sensation in the eyes and throat. Long-term exposure to formalin may also lead to skin disorders and cancer [14].

Direct Exposure to Body Fluids

Even though cadavers are disinfected by preserving them in embalming fluids, they can still carry several infections because the disinfection techniques that are being followed are not completely effective. As we deal with sharp instruments while dissecting, this can increase the chances of transmission of diseases such as HIV, hepatitis B, and tuberculosis through any cuts or open wounds on the skin of students or people handling cadavers that can accidentally happen during dissection [14].

Unhygienic Practices

Unprotected and improper clothing (laboratory coats), unclean hands, and instruments can act as carriers as various pathogens get lodged on them and can get administered into the body through any route [15].

Inadequate Ventilation and Ineffective Laboratory Practices

Several students working together in closed rooms/halls during dissection with improper ventilation can increase the chances of transmission of airborne diseases. Laboratory practices such as improper disposal of the dissection hall waste such as tissues and skin, inadequate disinfection, and preservation techniques of the cadavers are major risk factors for various disease transmission [15].

Specific body regions and the various bacterial species that are detected

According to the study that was conducted, specific regions of the body like the axilla, oral, nasal, and perineal regions of the cadavers were examined to check for the presence of bacteria [16]. The presence of skin folds in these regions makes them potential sites for the growth of bacteria. The particular regions of the sample collection are shown in Figure 1.

**Figure 1:** Specific regions of body chosen for bacterial detection. The image was taken by the author.

The identified bacterial species were further labeled as gram-positive or gram-negative species. The specific body region that they were identified from is mentioned in Table 1 [16].

**Table 1:** Bacteria cultured from the surfaces of formalin-fixed cadavers.

Bacterial species	Body region	Common infections caused
Aerococcus viridans	Axilla	Bacteraemia, endocarditis, urinary traction infections
Cellulomonas	Perineum	Bacteremia and catheter-related infections
Gardenerella vaginalis	Axilla	Bacterial vaginosis
Gemella hemolysans	Perineum	Eye infections, meningitis
Staphylococcus auricularis	Axilla	Skin and soft-tissue infections
Staphylococcus epidermidis	Axilla, oronasal, perineum	Bloodstream infections
*Staphylococcus haemolyticus*	Axilla, perineum	Bacteremia, meningitis, endocarditis
*Streptococcus mitis*	Oronasal	Dental and eye infections, infective endocarditis, bacteremia
Staphylococcus lugdunesis	Oronasal	Skin and soft-tissue infections, endocarditis
Corynebacterium striatum	Perineum	Bloodstream and catheter-related infections
Corynebacterium propinquum	Perineum	Infective endocarditis, respiratory tract infections
Kocuria varians	Oronasal	Urinary tract infections, peritonitis, bacteremia
Kocuria kristinae	Oronasal, perineum	Urinary tract infections
Gemella morbillorum	Axilla, oronasal	Infective endocarditis

A brief review of all identified bacterial species

Aerococcus viridians

These are gram-positive organisms that belong to the *Aerococcus *group and are considered contaminants that are seen in the hospital environment. *Aerococcus *was first described under a single species *A. viridans*; further, five more new species were identified, namely, *A. urinae*, *A. sanguinicola*, *A. christensenii*, *A. urinaehominis*, and *A. urinaeequi*. It is used as a source of lactate oxidase commercially. This is a gram-positive coccus and has a morphology similar to that of viridans streptococci. It is a rare pathogen that usually causes urinary tract infections, endocarditis, bacteremia, arthritis, or meningitis. *Aerococcus *shows fastidious growth and is usually confused with strains of *Streptococcus *and *Staphylococcus*. *Aerococcus *infections are usually treated by giving intravenous (IV) penicillin or ceftriaxone monotherapy [17].

Cellulomonas

It is a gram-positive, rod-shaped bacillus that has a special ability to degrade cellulose using specific enzymes such as endoglucanase and exoglucanase. They belong to the *Actinobacteria *group. This pathogen is also not very commonly seen, but it is recently noted to be one of the emerging pathogens for humans. Few cases have been reported where it caused endocarditis and osteomyelitis. Identification of cellulosomes on cadavers is unusual as it is usually found in soil and has cellulose activity. *Cellulomonas *strains usually possess various genes for the production of cellulases and xylanases [18].

Gardnerella vaginalis

The organism was named *Haemophilus vaginalis* when it was first identified. It is a facultative anaerobe that shows gram-variable staining because of the presence of a thin cell wall. These are non-motile and do not form spores. *Gardnerella *is normally found as a common organism of vaginal flora and contributes to maintaining balanced pH in the region. It causes bacterial vaginosis when it starts growing abnormally by involving other anaerobic bacteria and destroys the normal vaginal flora. It produces a toxin called vaginosis that affects human cells specifically [19].

Gemella hemolysins

It is a gram-positive, facultative anaerobe. They resemble *Neisseria *species. *Gemella *species are usually found in the oral cavity and respiratory tract of human beings where there is the presence of mucous membranes. *G. hemolysins* species is usually isolated from nasopharyngeal swabs of people. It is known to cause pulmonary exacerbations in patients with cystic fibrosis. The presence of this organism in the saliva is related to the periodontal health of the oral cavity and prevents the growth of *P. gingivalis* [20].

Staphylococcus auricularis

It is a gram-positive bacteria present in pairs or tetrads. This is usually found in the head region where abundant sebaceous glands are found, especially in the exterior region of the ear (auditory canal). It is weakly hemolytic. It is commonly found on human skin, causing sepsis or any other infections, but is usually a rare coagulase-negative *Staphylococci *(CoNS). Skin and soft-tissue infections are usually seen [21].

Staphylococcus epidermidis

It is a gram-positive bacteria and one of the common microflora that infects human epithelium. This typically belongs to human skin flora. The bacteria are usually found in hidden regions of the body and can cause boils and infections. It is an important opportunistic pathogen that gets easily attached to catheters and other medical devices to form biofilms. It is most commonly found in the axilla, head, and nostrils and belongs to the group of CoNS. These infections are usually treated with penicillin G, cephalosporins, etc. Vancomycin is used as the drug of choice for methicillin-resistant organisms [22].

Staphylococcus haemolyticus 

It is a gram-positive coccus and an opportunistic bacterial pathogen. It is usually found in the axilla, perineum, and inguinal regions and can cause bacteremia, meningitis, and skin or soft-tissue infections. This also has extreme antibiotic resistance and can be transmitted through direct or indirect contact with an infected person. *S. hemolyticus* can be rapidly inactivated through dry Cu. These infections are also usually hospital-acquired due to the administration of medical devices. The formation of biofilms makes the treatment of this bacteria more difficult. This organism also colonizes domestic animals [23].

Staphylococcus lugdunensis

It is a gram-positive bacteria that belongs to CoNS. They are usually hemolytic, appear in clusters, and have a sweet-smelling odor. It causes skin and soft-tissue infections such as cellulitis, cystic lesions, and peri-inguinal abscesses. It also causes a severe form of endocarditis, osteomyelitis, endocarditis, arthritis, and septicemia. It should be looked into for all routine investigations in the laboratories because they are one of the main pathogens for skin and soft-tissue investigations, especially in the groin region leading to cellulitis and abscesses [24].

Streptococcus mitis

*S. mitis* is gram-positive cocci that are spherical facultative anaerobe. It is an alpha-hemolytic species of *Streptococcus*. This bacteria was previously known as *S. mitior* and is usually found in the mouth, throat, nasopharynx, female genital tract, gastrointestinal tract, and skin. It has less virulence and pathogenicity but may cause severe infections such as endocarditis and meningitis which are life-threatening. Nearly 20 strains of *S. mitis* have been isolated from body fluids and are found to be susceptible to optochin. These bacteria move through the bloodstream to specifically get attached [25].

Corynebacterium striatum

This is a gram-positive, non-diptherial corynebacterium with a club-shaped morphology. They usually contaminate human skin and mucous membranes. They cause several infections including bacteremia, meningitis, pleuropneumonia, osteomyelitis, and uterine infections. It is one of the most emerging pathogens in various countries and is one of the most frequently isolated species of *Corynebacterium*. These bacterial infections are usually treated with monotherapy or amoxicillin-clavulanic acid in mild conditions, and in severe conditions, daptomycin or linezolid is used. It is a multi-drug-resistant pathogen that usually colonizes the nasopharynx [26].

Corynebacterium propinquum

It is a gram-positive aerobic bacteria that is normally a part of the oropharyngeal flora that is found in the skin and mucous membranes of the respiratory system. It is primarily isolated from the respiratory tract. It has been detected as a pathogen in infective endocarditis, prosthetic valve endocarditis, and nosocomial infections. These infections are usually seen in immune-compromised patients or those with underlying lung diseases. This can also cause other respiratory infections such as chronic obstructive pulmonary disease, bronchiectasis, and pneumonia. This species shows resistance to vancomycin and daptomycin. Proper identification of the species and the extent to which it could be pathogenic should be known to provide specific treatment [27].

Kocuria varians

It is a gram-positive bacteria that resembles *Staphylococcus *and *Micrococcus *and is arranged in pairs or tetrads. They are either aerobic or facultative anaerobic that have very rigid cell walls. It is generally found live on the skin and oral cavity. This bacteria is usually non-pathogenic but is related to specific infections such as urinary tract infections, cholecystitis, peritonitis, catheter-associated infections, brain abscess, and meningitis. *Kocuria *causes infections in immunosuppressed patients related to the oropharynx and deep cervical lymph nodes. These organisms grow on simple media plates or blood agar. They do not have the hemolytic ability on blood agar. *Kocuria *shows resistance to lysostaphin and nitrofurantoin [28].

Kocuria kristinae

It is a gram-positive bacteria that is formerly known as *Micrococcus kristinae*. This is normally found on human skin and oral mucosa and causes opportunistic infections. Recently, this organism was named *Rothia kristinae *after reclassifying the species. It is a facultative, non-motile anaerobe that forms pale cream to pale orange colonies on blood agar. *R. kristinae* is resistant to lysozyme. This organism is not considered to be a primary pathogen but is seen in patients under hospitalization, catheter-related bacteremia, patients undergoing dialysis, pregnant females, or patients with chronic illness. Treatment of this organism involves parenteral administration of vancomycin along with some other antibiotics [29].

Gemella morbillorum

It is a gram-positive coccus that lives in a microaerophilic environment. It was formerly known as *Streptococcus morbillorum*. It rarely causes any diseases, although it is found in the oropharyngeal area and gastrointestinal tract. *G. morbillorum* predominantly causes endocarditis, endovascular infections, and a few invasive infections. It is one of the most common bacteria found on teeth with cysts that do not get resolved even after repeated root canal treatments. These bacterial strains are usually resistant to penicillin. *G. morbillorum* has also been seen in colorectal cancer. It is one of the most common organisms to cause infective endocarditis in children. The most common cause of *G. morbillorum* is poor dental health or oral hygiene. It is a commensal of the upper respiratory tract of humans and gets into the bloodstream of patients to cause bacteremia [30].

Implications

This study helps us to know the presence of bacterial flora in different regions of the body, the importance of standard infection control methods that have to be followed by students and anatomists in the dissection hall to avoid the spread of any infections, and the need to improvise the dissemination methods that are currently being followed.

Proper clothing (laboratory coat), covering hair (using cap masks), hand gloves, table sterilization, proper disposal of unwanted tissues and debris after dissection, post-dissection hand washing and usage of hand sanitizers, and vaccination may prevent the spread of infections to some extent. The dissection hall should be maintained properly by proper cleaning with disinfectants such as phenol or formaldehyde. Covering the cadaver properly after usage with a sheet and disposing of all the waste as per the guidelines of biomedical waste management should be made compulsory. Hand washing limits the spread of the disease to a greater extent and should be well understood and followed by all the students and staff. Proper vaccination against hepatitis B, tuberculosis, etc. to avoid their transmission in accidental injuries while handling the cadavers is crucial.

As formalin also causes a lot of discomfort to students leading to watery eyes, dryness of mucous membranes, headache, nausea, and gastrointestinal disturbances, studies are ongoing to come up with better methods that can replace the usage of formalin or in alternate concentrations that can be completely effective for disinfection. It is required to look for an alternative to formalin as it is dangerous and hardens the tissues making dissection hard for students. Medical students, faculty members, and cadaver handlers who come in contact with cadavers in dissection halls are prone to get infected by these microorganisms. Formaldehyde fumes are harmful and cause skin and mucous membrane irritation. Researchers are now trying to identify different embalming procedures with a wide variety of chemicals instead of formalin. Above all, formalin is still used as a preservative and disinfectant in dissection halls because of its low cost, effectiveness, and results. Therefore, it is recommended to take proper precautions to avoid unnecessary exposure to chemicals and microorganisms until a proper alternative is identified.

## Conclusions

Numerous bacterial species have been identified in formalin-fixed cadavers that are given to medical students for dissection. For studying these bacteria, specific sites in the human body such as axillary, perineal, and oronasal regions were chosen as they are not usually contacted by people. These regions usually have skin folds that can prevent them from direct contact with formalin. Identification of bacterial flora will help us understand various kinds of diseases that can get transmitted to people dealing with cadavers. This clearly tells us the need to follow proper precautions while handling cadavers in dissection halls.
